RETRACTED

# Identification of Diagnostic Biomarkers of Rape Pollen Allergy Based on MRNA Sequencing

**DOI:** 10.1155/2022/6153577

**Published:** 2022-09-28

**Authors:** Jianhua Li, Fang Wang, Yunhua Cui, Li Song, Yongmei Yu, Xia Chen

**Affiliations:** ^1^Department of Otolaryngology, The Sixth Affiliated Hospital of Kunming Medical University, Yuxi, China; ^2^Department of Otolaryngology, The First Affiliated Hospital of Kunming Medical University, Kunming, China; ^3^Department of Pediatrics, Guandu District Maternal and Child Health Service Center, Kunming, China

## Abstract

In this study, 383 differentially expressed genes (DEGs) between the allergic group and the nonallergic group were excavated. Humoral immune response, chemokine-related biological processes, granulocyte-related biological processes, IL-17 signaling pathway, and TNF signaling pathway were found connected with DEGs. The allergic group had significantly higher enrich scores of T cells, T helper cells, TFH, and Th17 cells than the nonallergic group. We acquired 26 rape pollen allergy-associated genes by taking the intersection of key module genes from WGCNA and the DEGs. The functional enrichment results show that rape pollen allergy-associated genes are relevant to processes and pathways like regulation of inflammatory response, transcriptional regulation, lymphocyte differentiation, IL-17 signaling pathway, and MAPK signaling pathway. Then, three characteristic genes were defined by crossing the genes derived from LASSO and SVM-RFE algorithms, including *MYADM*, *PMAIP*1, and *MLF*1. The AUC values of these genes manifested that the three genes had a mighty discrimination power in discriminating allergic samples from nonallergic samples. In conclusion, this study revealed three characteristic genes (*MYADM*, *PMAIP*1, and *MLF*1) in rape pollen allergy, suggesting that they may be potential biomarkers in rape pollen allergy diagnosis and treatment.

## 1. Introduction

Allergic disease is mediated by one or more allergens I type hypersensitivity. Hay fever is one of the allergic diseases, which occurs after inhaling pollen allergens when the body contacts pollen allergen for the first time. The body produces IgE antibodies, combined in mast cells and basophils when the body contact with the same pollen allergen again. Pollen allergens and the cell surface of two or more than two adjacent IgE molecules bypass, mast cells degranulation, the release of a bioactive medium, cause itching, sneezing, nasal flow cleaning stuff, itchy eyes, nose, eye, and bronchial related symptoms such as cough, even can cause asthma, severely impair on the patient's quality of daily life. The incidence of hay fever is increasing year by year, and the reason is not clear. Rape pollen is airborne pollen, which can cause rape pollen allergy. Rape is one of the important oil and cash crops, and the rape flower has ornamental value. Due to its long flowering period, large pollen yield, and more contact with humans, rape pollen sensitization has been paid more and more attention.

RETRACTED

At present, the clinical diagnosis basis for rape pollen allergy is as follows: first, the patient has nasal itching, sneezing, and runny nose in spring, which can be accompanied by itching and coughing symptoms. Physical examination shows pallor and edema of the nasal mucosa, and the rape pollen skin prick test is positive. Rape pollen allergy desensitization mainly uses specific allergens, and this method gradually increases the dose to sensitize the allergic patients in a certain time interval to achieve a significant reduction of the corresponding symptoms when exposed to the allergen again. The efficacy of the treatment lasts for several years, but some patients relapse after treatment, and even a few patients have poorer treatment results [1]. Therefore, it is urgent to develop diagnostic biomarkers related to rape pollen allergy, explore the molecular mechanism of rape pollen allergy, and provide targets for disease treatment and diagnosis.

Based on transcriptomic second-generation high-throughput sequencing data from rape pollen allergic and nonallergic samples, this study revealed three characteristic genes (*MYADM*, *PMAIP*1, and *MLF*1) with diagnostic power, providing targets for disease treatment and diagnosis by bioinformatics approaches.

## 2. Materials and Methods

### 2.1. People and Sample Information

Peripheral blood mononuclear cell (PBMC) samples were collected from 8 cases of rape pollen allergy and 8 cases of nonrape pollen allergy in the Sixth Affiliated Hospital of Kunming Medical University, Yuxi, China. Samples are promptly reserved in liquid nitrogen to separate total RNA. All subjects gave informed consent. All specimens were collected and treated in accordance with the guidelines approved by the Ethics Committee of the Sixth Affiliated Hospital of Kunming Medical University (Approval No: kmykdx6f).

### 2.2. MRNA Sequencing

The total RNA of each sample was isolated using a Total RNA Purification Kit (TRK-1001, LC Sciences) on the basis of the manufacturer's protocols. Total RNA was quantitated on a NanoDrop ND-2000 (Thermo Scientific), and the RNA integrity was measured using an Agilent Bioanalyzer 2100 (Agilent Technologies). The construction of the next-generation sequencing libraries and sequencing were executed by LC-bio Technologies co., ltd (Hangzhou, China). The transcriptome clean data were obtained and aligned with the human genome (hg19) in the HISAT2 software [2]. SAMtools was used to sort reads in binary alignment map (bam) file by chromosome [3]. Then we used the featureCount program to count the reads and quantify mRNA [4].

RETRACTED

### 2.3. Identification of Differentially Expressed Genes (DEGs)

The differentially expressed genes (DEGs) between the allergic group (case) and nonallergic group (control) were determined by the “DEseq2” R package [5]. The log_2_ Fold Change (FC)| ≥ 1 and *P* value < 0.05 were deemed as the threshold value for DEGs. A volcano map was plotted to present the distinction in gene expression levels between the two groups. A heatmap was plotted to display the expression of the top 50 DEGs.

### 2.4. Functional and Pathway Enrichment Analysis

The “clusterProfiler” R package was employed to execute GO and KEGG analysis [6]. The criterion for enrichment significance was *P* value < 0.05. GO enrichment analysis specified the biological processes (BP), cellular components (CC), and molecular functions (MF) relevant to DEGs. KEGG pathway analysis uncovered biological pathways connected with DEGs. To further uncover the signaling pathways in which DEGs between two groups were enriched, gene set enrichment analysis (GSEA) was also implemented employing the “c2.cp.kegg.v7.4.symbols.gmt” gene set as a reference gene set.

### 2.5. Immune Cell Infiltration Analysis

The enrichment fraction of 23 immune cells in each sample was calculated by the single-sample gene set enrichment analysis (ssGSEA) algorithm [7]. The box plot and heatmap were drawn to manifest the distinction in 23 immune cells infiltration between the allergic group (case) and the nonallergic group (control).

### 2.6. Weighted Gene Coexpression Network Analysis (WGCNA)

The transcriptome data of 8 samples allergic to rape pollen (case) and 8 control samples (control) was analyzed by the “WGCNA” R package [8]. The “goodSamplesGenes” function was used to filter out low expressing genes and perform sample clustering to identify and remove outliers. For making the coexpression network contented with the distribution of a scale-free network, the pickSoftThreshold function was utilized for computing the soft-thresholding power. The dynamic tree cutting method was used to identify different modules. Then, we set a merging threshold of 0.4 to merge similar modules. The correlation between the modules and two clinical traits (control and case) was further analyzed. Finally, the module with the highest Pearson correlation coefficient was chosen for subsequent analysis.

### 2.7. Diagnostic Genes Screening and Verification

The least absolute shrinkage and selection operator (LASSO) is an algorithm that can be used to obtain a more sophisticated model by structuring a penalty function [9]. Support vector machine–recursive feature elimination (SVM-RFE) is a support vector machine-based characteristic selection algorithm that ranks characteristics based on recursive feature deletion sequences [10]. LASSO and SVM-RFE algorithms were utilized to identify the diagnostic genes in rape pollen allergy by the “glmnet” and “e1071” packages, respectively. Crossed genes screened by two algorithms were regarded as diagnostic genes. The area under the curve (AUC) value of receiver operating characteristic (ROC) was utilized to determine the diagnostic effectiveness of potential biomarkers in discriminating rape pollen allergic samples from normal samples and performed by using the pROC package [11].

RETRACTED

### 2.8. Statistical Analysis

Whole analyses were conducted using the R language, and the data from different groups were compared by the Wilcoxon test. If not specified above, a *P* value less than 0.05 was taken as statistically significant.

## 3. Results

### 3.1. Functional and Pathway Enrichment Based on the DEGs between the Rape Pollen Allergic Group and Rape Pollen Nonallergic Group

Firstly, 383 DEGs, including 232 upregulated genes and 151 downregulated genes between the rape pollen allergic group and rape pollen nonallergic group, were excavated (Figure 1(a), Table S1). The expressions of the top 50 DEGs were presented in Figure 1(b). Then, 75 GO items, including 51 BP items, 19 MF items, 5 CC items, and 17 KEGG pathways were enriched based on DEGs (Table S2). The top 10 terms in BP, MF, and the significant CC terms were listed in Figure 1(c). We noted that allergy-related GO terms, including chemokine-mediated signaling pathway, response to chemokine, granulocyte chemotaxis, granulocyte migration, and humoral immune response in BP, chemokine activity, immunoglobulin binding, and chemokine receptor binding in MF were enriched. Meanwhile, 17 enriched KEGG pathways were revealed in Figure 1(d). Among them, cytokine-cytokine receptor interaction, IL-17 signaling pathway, chemokine signaling pathway, and TNF signaling pathway were found related to DEGs between the rape pollen allergic group and rape pollen nonallergic group. We further performed GSEA based on transcriptome data of the rape pollen allergic group and rape pollen nonallergic group and the results revealed that 17 KEGG pathways were enriched, including cytokine–cytokine receptor interaction and chemokine signaling pathway (Table S3). Top 10 pathways were displayed in Figure 1(e).

### 3.2. The Differential Immune Cell between the Rape Pollen Allergic Group and Rape Pollen Nonallergic Group

The functional and pathway enrichment results suggested that immune-related biological processes and pathways were related to rape pollen allergy. To explore the discrepancy in immune cells between the rape pollen allergic group and the rape pollen nonallergic group, we estimated the fractions of 23 immune cells of each sample using the ssGSEA algorithm. As shown in Figures 2(a) and 2(b), the rape pollen allergic group had notably higher enrich scores of T cells, T helper cells, TFH, and Th17 cells than the rape pollen nonallergic group and the rape pollen nonallergic group had significantly higher enrich scores of Macrophages and Tgd than the allergic group. The difference in the relative mean infiltrating score of the same immune cell in the two groups was shown in Figure 2(c). Then, we analyzed the Pearson correlation between each immune cell to inspect their relationship and probable interaction. As revealed in Figure 2(d), among all immune cells, T cells possessed the highest correlation with T helper cells (Pearson's correlation = 0.92), and the second greatest positive correlation was the relevance between Th17 cells and T helper cells (Pearson's correlation = 0.79). Moreover, macrophages showed a powerful negative correlation with both T cells and T helper cells (Pearson's correlation = −0.75, −0.74).

RETRACTED

### 3.3. Identification of Genes Associated with Rape Pollen Allergy

To excavate the key modules most associated with rape pollen allergy, we structured WGCNA on the genes in the transcriptome data of the rape pollen allergic group and rape pollen nonallergic group. No obvious outlier samples were removed by clustering and *β* = 9 (scale-free *R*^2^ = 0.85) was selected to construct a scale-free network (Figure 3(a) and 3(b)). Then, a cluster dendrogram was constructed and a dynamic tree cut was performed. 23 modules were obtained and 19 modules were eventually developed after merging (Figures 3(c) and 3(d)). Subsequently, we assessed the correlation of each module with two clinical traits. The results indicated that the MEred module (cor = 0.88, *P* = 0.000006) had the highest correlation with rape pollen allergy (Figure 3(e)). Thus, we extracted 200 key module genes from the module with MM > 0.8 and GS > 0.2 for further analysis (Figure 3(f), Table S4). Finally, we acquired 26 rape pollen allergy-associated genes by overlapping 200 key module genes and the 383 DEGs between the rape pollenallergic group and rape pollen nonallergic group (Figure 3(g), Table S5).

Next, we performed GO and KEGG enrichment analysis on 26 rape pollen allergy-associated genes. 174 GO items, including 167 BP items, 2 MF items, 5 CC items, and 5 KEGG pathways were enriched (Table S6, Figure 4(a) and 4(b)). Top 10 BP terms were shown in Figure 4(a). Among the enriched terms, rape pollen allergy-associated genes were significantly related to the regulation of transcription from RNA polymerase II promoter in response to stress, positive regulation of transcription regulatory region DNA-binding, regulation of leukocyte differentiation, regulation of ERK1 and ERK2 cascade, regulation of regulatory T cell differentiation, regulation of lymphocyte differentiation, leukocyte activation involved in an inflammatory response, regulation of inflammatory response, regulation of cytokine secretion, positive regulation of cytokine production, and regulation of DNA-binding transcription factor activity in BP. Concerning KEGG pathways, rape pollen allergy-associated genes were engaged in the IL-17 signaling pathway, apoptosis, and MAPK signaling pathway.

RETRACTED

### 3.4. Identification of Characteristic Genes in Rape Pollen Allergy

We analyzed the Pearson correlations of 26 rape pollen allergy-associated genes with differential immune cells between the rape pollen allergic group and rape pollen nonallergic group. The pairs with *P* value < 0.05 and |correlation coefficient > 0.3 were retained and visualized using cytoscape (Table S7, Figure 5(a)). Then, we selected 23 genes with a high correlation with differential immune cells out of 26 genes (*P* value < 0.05 and |correlation coefficient > 0.6, Table S8).

To screen characteristic genes from the 23 genes, we employed LASSO and SVM-RFE algorithms. Four characteristic genes (*MYADM*, *CFAP*20, *PMAIP*, and *MLF*1) were discerned using the LASSO algorithm (Figure 5(b)). The ROC curve of the LASSO regression model was plotted and the AUC value = 1, indicating the model based on the four characteristic genes could distinguish rape pollen allergic samples and rape pollen nonallergic samples accurately (Figure 5(c)). In the meantime, seven characteristic genes (*MLF*1, *DUSP*10, *PMAIP*1, *CYP2F*1, *KLF*4, *MYADM*, and *KIF*9) were picked with the SVM-RFE algorithm, as exhibited in Figures 5d1-5d2. Three characteristic genes were determined by crossing the genes extracted from these two algorithms, including *MYADM*, *PMAIP*1, and *MLF*1 (Figure 5(e)). The logistic regression model was constructed based on three characteristic genes. The AUC value of the ROC curve was 1 (Figure 5(f)). Then, we plotted the heatmap to illustrate the predictive ability of the logistic regression model, LASSO model, and SVM model (Figure 5(g)). Finally, we evaluated the diagnostic value of each characteristic gens by ROC analysis. The AUC values of these genes were all 1, suggesting that *MYADM*, *PMAIP*1, and *MLF*1 had a powerful discrimination ability in discriminating allergic samples from nonallergic samples (Figure 5(h)).

RETRACTED

## 4. Discussion

Rape pollen allergy can cause symptoms related to the nose, eyes, and bronchus. At present, diagnosis of rape pollen allergy mainly depends on history, physical examination, and skin prick test. The specific allergen desensitization therapy is used in treatment, but this method still cannot completely block the occurrence and development of allergic diseases and cannot completely cure them.

Based on differential gene screening and functional enrichment, we found that chemokine-related biological processes, granulocyte-related biological processes, and humoral immune processes were related to differential genes. Il-17 signaling pathway and TNF signaling pathway were also enriched. Rape pollen allergy belongs to humoral immunity. Studies have revealed that these biological processes are involved in the incidence and progression of allergic rhinitis [12]^.^ Il-17 is a characteristic cytokine secreted by Th17 cells, and the TH17-IL-17 axis is now known to play an important role in host defense, the pathogenesis of autoimmune diseases, and tumors. Related studies have reported that TNF-A is released by activated mononuclear macrophages, which can play a part in regulating the body's immune response, while NF-KB exerts a notable role in allergic diseases, also participates in the regulation of TNF-A and plays a crucial role in the pathogenesis of AR [13].

The results of functional enrichment indicated that immune-related processes and pathways were related to rape pollen allergy. Therefore, based on the analysis of transcriptomic data and the ssGSEA algorithm, we found that there was higher infiltration of T cells, T helper cells, TFH, and Th17 cells in the sensitive group. TFH secretes IL-21 and expresses CD40L and other membrane molecules which act on B cells and exert a key role in the development of germinal centers and the formation of plasma cells. TFH secretes IL-21, IL-4, or IFU-r by expressing CD40L and participates in the class conversion of antibodies. CD40L can stimulate B cells. Participating in the selection process of high-affinity B cells, TFH can also regulate the function of memory B cells and promote their ability to generate and maintain immune responses in the long term. Th17 plays a notable part in the occurrence and progress of innate immunity and certain inflammation by secreting various cytokines such as IL-17, IL-21, IL-22, IL-26, and TNF-*α* [14], among which IL-17 can stimulate local tissue cells to produce chemokines and cytokines such as G-CSF, and recruit neutrophils and monocytes. By stimulating neutrophil hyperplasia and activation, IL-22 can contribute to tissue damage and inflammatory diseases by stimulating epithelial cells to secrete chemokines and other cytokines. Il-21 can stimulate the proliferation, differentiation, and effect of CD8+T cells and NK cells through paracrine stimulation and amplification of TH17 function, and participate in the immune response of B cells [15]. Rape flower powder allergy is the humoral immune response responsible for B cells, and cells enriched in the sensitive group exert an important part in the allergic reaction. Based on WGCNA and differential genes, we obtained 26 genes related to pollen allergy in rape flowers. Through functional enrichment results, we learned that these genes were related to inflammatory response regulation, transcriptional regulation, lymphocyte differentiation, and other processes, as well as the IL-17 signaling pathway and MAPK signaling pathway. Il-17 is a proinflammatory cytokine secreted by Thl7 cells and has a variety of biological activities. Studies have found that IL-17 can play a role by stimulating the release of inflammatory cytokines from target cells and the cytokines regulating neutrophils, inducing the production of B-6, NO, and prostaglandin E2, and simultaneously upregulating the expression of inflammatory cytokines like Y-interferon, TNF-A, and CD40 ligand, promoting the incidence and development of local inflammation [16]. MAPK pathway exerts a crucial role in cell proliferation, differentiation, stress, inflammation, functional synchronization, transformation, apoptosis, and other signal transduction pathways. Mitogen-activated protein kinase (MAPK8), MAPK1, and MAPK14 are all members of the MAPK family. MAPK is one of the vital signal transduction systems in organisms, which can be activated by various inflammatory stimuli and acts as an important regulator in the genesis and development of inflammation [17]. In T cells, *MAPK*8 and *MAPK*9 are required for Th cells to differentiate into Th1 cells. Animal experiments showed that *MAPK8* knockout mice relieved the symptoms of atopic dermatitis [18]. *MAPK*1/*ERK*2 and *MAPK*3/*ERK*1 are the two maps to be involved in the *MAPK*/*ERK* cascade. Erk1/2 is associated with allergic inflammation involving Th2 differentiation and proliferation. Phosphorylation of *ERK1*/2 *MAPK* in the airways causes inflammation and structural changes that lead to T cell activation, eosinophils and mast cell infiltration, bronchial hyper-reactivity, and airway remodeling [19]. *MAPK*14/P38 *α* regulates several T cell receptor-related signals and affects Th2 differentiation and allergic inflammation negatively [20]^.^*MAPK* is closely related by participating in inflammation, cell differentiation, stress, and inflammatory response related to rape allergy. Meanwhile, the IL-17 family activates anticytokines and chemokines in the MAPK pathway. Through correlation analysis, we obtained 23 genes highly correlated with the differential immune cells, and these results provide information for further research on the function of these genes. Based on 23 genes, 3 characteristic genes were screened by machine learning method, and 3 characteristic genes had a good diagnostic ability, which could distinguish rape pollen allergy samples from nonallergic samples. *MYADM* is a marker of myeloid-related differentiation. It has been found that *MYADM* is a MAL family protein that regulates endothelial barrier function and the function and dynamics of organized membrane domains [21].

RETRACTED

Phorbol-12-myristate-13-acetate-induced protein 1 (PMAIP1), a Bcl-2 homology domain 3 (BH3)-only protein, is a p53-derivable gene that is responsive to DNA damage [22]. PMAIP1 enables Bak/Bax release, which enables it to bind to antiapoptotic Mcl-1 and A1, thus serving a pro-apoptotic function [23]. Furthermore, a changed expression of PMAIP1 has been noted in multiple cancers, including colorectal carcinoma, breast carcinoma, and endometrial carcinoma [24]. Myeloid leukemia factor 1 (MLF1) is a protein engaged in myeloid cell differentiation which regulates the cell cycle and the expression of numerous genes. The MLF1 gene codes for a 30 kDa intracellular protein that is most commonly known for its role in regulating the commitment of hematopoietic progenitor cells into the myeloid lineage and restricting erythroid formation [25]. MLF1 interacts with a number of other proteins and is thought to act as a transcription factor due to its DNA-binding domains and ability to modulate gene expression. Many of the normal functions of *MLF*1 involve cell cycle regulation [26]. In cancer, translocations of the *MLF*1 gene and the nucleophosmin gene have been associated with acute myeloid leukemia and myelodysplastic syndrome [27]. Until now, there are no relevant reports on the studies of these three genes in rape pollen allergy. This is the first time that we found that these three genes are characteristic genes of rape pollen allergy and have the diagnostic ability. These three genes are highly correlated with Th17 cells and TFH, and their mechanism of action in rape pollen allergy needs further research.

Although we identified three signature genes (*MYADM*, *PMAIP*1, and *MLF*1) for the diagnosis of rape pollen allergy, there still have some limitations in our study. First, the sample size limitations may bias our results, more samples with rape pollen allergy information were needed to be included in the study and confirm the reliability of our study. Secondly, we explored the functions of these three signature genes only through a series of bioinformatics analyses, and experimental data were needed to support these conclusions. Despite these limitations, this study adopted the ROC curve to demonstrate the prognostic predictive validity of the three signature genes.

RETRACTED

## Figures and Tables

**Figure 1:** Functional and pathway enrichment based on the DEGs between the rape pollen allergic group and rape pollen nonallergic group. (a) The volcano graph of DEGs, (b) the heat map of DEGs, (c) the bubble plot of TOP 10 GO items in BP, CC, and MF category, (d) the bar plot of enriched KEGG pathways, (e) top 10 KEGG pathways enriched by GSEA.

**Figure 2:** Immune cell infiltration profiling. (a) The differential immune cells analysis by ssGSEA. (b) The heatmap of immunocyte. (c) The relative percentage of immune cells. (d) Pearson correlation between immune cells.

**Figure 3:** Weighted gene coexpression network analysis. (a) Sample cluster, (b) the determination of soft threshold, (c) cluster dendrogram to merge similar modules, (d) the cluster dendrogram of coexpression modules, (e) the correlation between modules and clinical traits, (f) correlation of genes within modules with models and traits, (g) the overlapping of key module genes and DEGs.

**Figure 4:** Functional enrichment of genes associated with rape pollen allergy. (a) The enriched top 10 GO (BP) terms, GO (CC) terms, and GO (MF) terms. (b) The bar plot of enriched KEGG pathway.

**Figure 5:** Identification of characteristic genes in rape pollen allergy. (a) The correlation between differential immune cells and rape pollen allergy-related genes, (b) the LASSO regression analysis, (c) the ROC curve of LASSO regression model, D1-2, (d) the SVM analysis, (e) the intersection of characteristic genes authenticated by LASSO and SVM, (f) the ROC curve of the logistic regression model, (g) the ROC curves of characteristic genes, (h) the heatmap of each model's ability to predict samples.

## Data Availability

Some or all data, models, or code generated or used during the study are available from the corresponding author by request.

## Supplementary Materials

Supplementary Materials Table S1: DEGs between the rape pollen allergic group and rape pollen nonallergic group. Table S2: Enriched GO items and KEGG pathways of DEGs by ClusterProfiler. Table S3: Underlying KEGG pathways of DEGs by GSEA. Table S4: Genes in MEred module. Table S5: Rape pollen allergy-associated genes between DEGs and key module genes. Table S6: Enriched GO items and KEGG pathways of rape pollen allergy-associated genes. Table S7: Correlations of rape pollen allergy-associated genes with differential immune cells between the rape pollen allergic group and rape pollen nonallergic group. Table S8: Rape pollen allergy-associated genes with high correlation with differential immune cells.

RETRACTED

## References

[1] Subspecialty Group of Rhinology Editorial Board of Chinese Journal of Otorhinolaryngology Head and Neck Surgery (2011). Expert consensus on allergen specific immunotherapy of allergic rhinitis. *Zhonghua Er Bi Yan Hou Tou Jing Wai Ke Za Zhi*.

[2] Kim D., Paggi J. M., Park C., Bennett C., Salzberg S. L. (2019). Graph-based genome alignment and genotyping with hisat2 and hisat-genotype. *Nature Biotechnology*.

[3] Li H., Handsaker B., Wysoker A. (2009). The sequence alignment/map format and samtools. *Bioinformatics*.

[4] Liao Y., Smyth G. K., Shi W. (2014). Featurecounts: an efficient general purpose program for assigning sequence reads to genomic features. *Bioinformatics*.

[5] Love M. I., Huber W., Anders S. (2014). Moderated estimation of fold change and dispersion for rna-seq data with deseq2. *Genome Biology*.

[6] Yu G., Wang L. G., Han Y., He Q. Y. (2012). Clusterprofiler: an r package for comparing biological themes among gene clusters. *Omics-a Journal of Integrative Biology*.

[7] Bindea G., Mlecnik B., Tosolini M. (2013). Spatiotemporal dynamics of intratumoral immune cells reveal the immune landscape in human cancer. *Immunity*.

[8] Langfelder P., Horvath S. (2008). WGCNA: an r package for weighted correlation network analysis. *BMC Bioinformatics*.

[9] Friedman J., Hastie T., Tibshirani R. (2010). Regularization paths for generalized linear models via coordinate descent. *Journal of Statistical Software*.

[10] Huang M. L., Hung Y. H., Lee W. M., Li R. K., Jiang B. R. (2014). Svm-rfe based feature selection and taguchi parameters optimization for multiclass svm classifier. *The Scientific World Journal*.

[11] Robin X., Turck N., Hainard A. (2011). Proc: an open-source package for r and s+ to analyze and compare roc curves. *BMC Bioinformatics*.

[12] Li H.. , L., Duan Z.. , J. (2018). Research progress of allergic rhinitis. *Inner Inner Medicine Journal*.

[13] Zhaonan M. A., Wang J., Yan M. A., Wang S. (2017). Exploring the effect of xiaoqinglong decoction and yupingfeng powder on the content of tnf-*α* and the expression of tnf-*α* mrna in rats with allergic rhinitis based on nf-*κ*b signaling pathway. *Journal of Liaoning University of Traditional Chinese Medicine*.

[14] Cao X. T. (2018). *Medical Immunology*.

RETRACTED

[15] Cao X. T. (2018). *Medical Immunology*.

[16] Marcal J. R. B., Samuel R. O., Fernandes D. (2010). T-helper cell type 17/regulatory t-cell immunoregulatory balance in human radicular cysts and periapical granulomas. *Journal of Endodontics*.

[17] Jiang Y., Gong X.. , W. (2000). Regulation of inflammatory responses by MAPK signal transduction pathways. *Sheng Li Xue Bao*.

[18] Choi J., Kim J. R., Kim H. (2013). The atopic dermatitis-like symptoms induced by mc903 were alleviated in jnk1 knockout mice. *Toxicological Sciences*.

[19] Dandekar R. D., Khan M. M. (2011). Regulation of ERK2 phosphorylation by histamine in splenocytes. *Immunopharmacology and Immunotoxicology*.

[20] Hu P., Nebreda A. R., Liu Y., Carlesso N., Kaplan M., Kapur R. (2012). P38*α* protein negatively regulates t helper type 2 responses by orchestrating multiple t cell receptor-associated signals. *Journal of Biological Chemistry*.

[21] Aranda J. F., Reglero-Real N., Marcos-Ramiro B. (2013). Myadm controls endothelial barrier function through erm-dependent regulation of icam-1 expression. *Molecular Biology of the Cell*.

[22] Zhao X., Liu X., Su L. (2014). Parthenolide induces apoptosis via tnfrsf10b and pmaip1 pathways in human lung cancer cells. *Journal of Experimental & Clinical Cancer Research*.

[23] Idrus E., Nakashima T., Wang L. (2011). The role of the bh3-only protein noxa in bone homeostasis. *Biochemical and Biophysical Research Communications*.

[24] Kapoor S. (2008). Altered expression of the pmaip1 gene: a major player in the evolution of gastrointestinal and systemic malignancies. *Digestive Diseases and Sciences*.

[25] Ota T., Suzuki Y., Nishikawa T. (2004). Complete sequencing and characterization of 21, 243 full-length human cdnas. *Nature Genetics*.

[26] Yoneda-Kato N., Tomoda K., Umehara M., Arata Y., Kato J. Y. (2005). Myeloid leukemia factor 1 regulates p53 by suppressing cop1 via cop9 signalosome subunit 3. *The EMBO Journal*.

[27] Yoneda-Kato N., Look A. T., Kirstein M. N. (1996). The t(3;5)(q25.1;q34) of myelodysplastic syndrome and acute myeloid leukemia produces a novel fusion gene, npm-mlf1. *Oncogene*.

